# A compact photometer based on metal-waveguide-capillary: application to detecting glucose of nanomolar concentration

**DOI:** 10.1038/srep10476

**Published:** 2015-05-28

**Authors:** Min Bai, Hui Huang, Jian Hao, Ji Zhang, Haibo Wu, Bo Qu

**Affiliations:** 1 Department of Electronic Science and Technology, Faculty of Electronic Information and Electrical Engineering, Dalian University of Technology, Dalian 116024, China; 2 Jordan Valley Semiconductors UK Ltd, Shanghai 201206, China

## Abstract

Trace analysis of liquid samples has wide applications in life science and environmental monitor. In this paper, a compact and low-cost photometer based on metal-waveguide-capillary (MWC) was developed for ultra-sensitive absorbance detection. The optical-path can be greatly enhanced and much longer than the physical length of MWC, because the light scattered by the rippled and smooth metal sidewall can be confined inside the capillary regardless of the incident-angle. For the photometer with a 7 cm long MWC, the detection limit is improved ~3000 fold compared with that of commercial spectrophotometer with 1 cm-cuvette, owing to the novel nonlinear optical-path enhancement as well as fast sample switching, and detecting glucose of a concentration as low as 5.12 nM was realized with conventional chromogenic reagent.

Photometry is widely used for trace analysis of liquid samples, because abundant chromogenic reagents and semiconductor optoelectronic devices are available^1^,^2^,^3^,^4^,^5^. In comparison with conventional cuvette-based absorbance detection, liquid waveguide capillary (LWC) can provide long optical-path (up to several meters) for ultra-sensitive detection while retaining small sample volume, by confining the probe light inside the capillary via total internal reflection (TIR)^1^,^2^,^3^,^4^,^5^. However, the optical-path is only nearly equal to the physical length of LWC without further enhancement^3^,^6^, and increase of LWC length longer than 1.0 m would suffer from high attenuation of light and high risk of gas bubble formation, etc^3^,^7^. As for the multi-reflection cell, which was proposed for optical-path enhancement, the improvement on detection limit is only 2.5 fold^8^,^9^.

Currently, there are mainly two kinds of LWC, i.e., Teflon AF capillary (whose refractive-index is only ~1.3 and less than that of water), silica capillary coated with Teflon AF or metal films^1^,^3^,^4^. The low refractive-index material and large light incident-angle are required for realizing TIR at interface of dielectric materials^3^,^6^,^10^. As for Teflon AF capillary, Teflon AF is permeable to gas and could absorb little species in aqueous sample, due to its porous structure^3^,^11^. For silica capillary externally coated with Teflon AF or metal, the light tends to be guided in the silica cladding layer rather than in the liquid core, because the refractive-index of silica (1.45) is higher than that of most liquid samples (e.g. 1.33 for water)^3^,^6^,^12^,^13^. As for the capillary internally coated with metal film, the transmitting characteristics have been investigated^14^,^15^,^16^,^17^,^18^, but the coating process is complicated and the metal film suffers from the rough surface and porous structure^4^,^19^.

Moreover, for the commercial LWC (Teflon AF capillary and Teflon AF coated silica capillary, World Precision Instruments, Inc), they still have some other shortcomings, such as (1) capillary bending could make the light leak out of capillary due to the failure of TIR^3^,^10^, (2) large dead volume in T-connector (which is used for connecting the capillary, optical fiber and inflow/outflow pipe) could trap gas bubbles^10^.

Meanwhile, glucose detection is important for diagnosing diabetes mellitus, hepatocirrhosis and psychopathy, etc^20^., and many detection methods, such as photometry (including spectrophotometry^21^,^22^,^23^,^24^,^25^ and paper based colorimetry^26^,^27^,^28^), amperometry^29^,^30^,^31^, fluoremetry^32^,^33^,^34^,^35^, polarimetry^36^, surface plasmon resonance^37^, Fabry-Pérot cavity^38^, electrochemistry^39^, and capillary electrophoresis^40^,^41^ etc., have been reported. However, most of these methods require expensive equipments and detecting glucose of a few nanomolar concentration is still a challenge (e.g., for photometry measurement^21^,^22^,^23^,^24^,^25^,^26^,^27^,^28^, till now the lowest detection limit of glucose is only 30 nM by using Prussian blue nanoparticles as peroxidase mimetics^21^). For the cell researches on molecular level, nanomolar glucose detection is normally required, such as inhibitive growth of human prostate cancer^42^ and CO_2_ fixation behaviors of Prochlorococcus in the Ocean^43^.

In this paper, a compact and low-cost photometer based on metal-waveguide-capillary (MWC), which is a SUS316L stainless steel capillary with electropolishing internal surface, was developed for ultra-sensitive absorbance detection. Because light can be confined inside the metal capillary regardless of the incident-angle, the optical-path can be greatly enhanced and much longer than the physical length of MWC, via light scattering at the rippled and smooth metal surface. Moreover, for optical coupling and fluid inlet/outlet, a simple T-connector was developed to minimize the dead volume and avoid gas bubble trapping. For the photometer with a 7 cm long MWC, the detection limit is improved ~3000 fold compared with that of commercial spectrophotometer with 1cm-cuvette, owing to the novel nonlinear optical-path enhancement as well as fast sample switching, and detecting glucose of a concentration as low as 5.12 nM was realized with conventional chromogenic reagent.

## Results and discussions

### Performance of MWC-based photometer

As shown in Fig. 1, the MWC-based photometer consists of a 7cm long MWC with EP grade electropolishing inner surface, a 505 nm LED with a lens, a gain tunable photodetector, and two T-connectors used for optical coupling and fluid inlet/outlet. A three-way valve connected to the inlet Peek pipe is used to switch the inflow samples. The Peek pipe is close with the quartz plate and MWC, so the dead volume in the T-connector can be minimized to effectively avoid gas bubble trapping. Moreover, the collimated light beam can be easily and efficiently coupled into the MWC through the quartz plate of T-connector.

The light beam and the liquid sample were introduced into the MWC via the T-connector, and the beam transmitting through the MWC was received by the photodetector. The inflow solution of the *colored-* or *blank-sample* was introduced alternately into the MWC via the three-way valve. According to Beer’s law, the absorbance of *colored-sample* can be calculated via Eqs. 1.^10^

Where *V*_*color*_ and *V*_*blank*_ are output signals of the photodetector when the *colored-* and *blank-samples* are introduced into the MWC, respectively, and *V*_*dark*_ is the background signal of the photodetector when the LED is turned off. The output signal variation *ΔV = V*_*color*_ *– V*_*blank*_ can be measured by switching samples. According to Eqs. 1, if *ΔV* is much smaller than *V*_*blank*_–*V*_*dark*_, slight variation in *V*_*blank*_ (e.g., signal drifting) has a negligible effect on *A*_*MWC*_ value by using the sample switching scheme.

In order to compare the performance of MWC-based photometer with that of cuvette-based spectrophotometer, red-ink solution was used as *colored-sample* due to its excellent color stability and good linearity in concentration-absorbance relationship, and DI H_2_O was used as *blank-sample*. As shown in Table 1, a series of red-ink solutions were prepared with DI H_2_O as solvent by using successive dilution method. The relative concentration of sample 1 (S1), which is original red-ink without dilution, is defined as 1.0. Figure 2 shows the optical photograph of the eleven red-ink samples (from S4 to S14) with relative concentrations (as listed in Table 1) ranging from 8.0 × 10^-3^ (on left) to 8.2 × 10^-10^ (on right).

The measurement result of sample 6 is shown in Fig. 3(a). The time, when switching takes place between the *colored-* and *blank-samples*, is marked by double arrow “↔” in the figure. It is clear that the output voltage increases rapidly when switching from *colored-* to *blank-sample*, and it decreases vice versa. The *V*_*color*_, *V*_*blank*_ and corresponding *ΔV* can be obtained as shown in the figure.

The measurement results of sample 9, 13 and 14 are shown by Fig. 3(b)–(d), respectively. As shown in Fig. 3 (d), the measured *ΔV* is only 5 nV, which is nearly 3 times of the noise value (2 nV). Smaller *ΔV* is hard to be discriminated from the noise. Thus, the detection limit reaches a relative concentration of 8.2 × 10^-10^ (sample 14). By using Eqs. 1, the absorbance *A*_*MWC*_ can be calculated with the measured *V*_*color*_, *V*_*blank*_ and *V*_*dark*_. The *V*_*dark*_ is −0.68 μV for the photodetector with an amplification-factor of 10^4^. Measurement results of all samples were summed up in Table 1 and can be founded in supplemental material. As indicated in Table 1, the detected absorbance becomes saturated at high concentration, so the absorbance larger than 3.7 can not be measured by using the MWC-based spectrometer.

For comparison, the red-ink samples were also measured by using the spectrophotometer, and the measured absorbance *A*_*cuvette*_ are shown in Fig. 4. The values of *A*_*cuvette*_ at 505 nm (as listed in Table 1) was obtained by regarding the curves of sample 10, 11, or 12 (as shown by the inset of Fig. 4) as the baseline. As shown in the figure, the detection limit reaches a relative concentration of 2.56 × 10^-6^ (sample 9), because the absorbance curves of sample 10, 11 and 12 can not be discriminated from each other. Thus, in comparison with the cuvette-based spectrophotometer, a 3125-fold improvement on detection limit was achieved by using the MWC-based photometer.

The absorbance-concentration relationship was plotted in Fig. 5. For the cuvette-based measurement, the absorbance is proportional to the ink concentration with a constant optical-path of 1 cm. While for the MWC-based measurement, nonlinear enhancement in absorbance is observed at low concentrations. According to Beer’s law, absorbance is proportional to the optical-path, so the absorbance-enhancement-factor AEF (defined as AEF *= A*_*MWC*_*/A*_*cuvette*_ at the same ink concentration) is the ratio between the optical-path of the MWC and cuvette. As shown in Fig. 5, at high concentrations, AEF has a constant value of ~7.0, which is reasonable because the length of MWC is exactly 7 times that of 1 cm cuvette. However, at low concentrations (related concentration <1.28 × 10^-5^ ), AEF increases with decreasing concentration and would reach a value of 803 at related concentration of 8.2 × 10^-10^ by extrapolating the curve of cuvette-based measurement. Thus, the corresponding optical-path as long as 803 cm (AEF×1 cm) can be obtained, which is much longer than the physical length of MWC and even longer than the commercial longest LWC (500 cm long for World Precision Instruments, Inc, and 200 cm long for Doko Engineering LLC). This nonlinear enhancement of absorbance in LWC has not been reported previously.

### Analysis and discussion

Fig. 6(a)–(c) show the optical image, microscopy image and optical surface profiler image, respectively, of inner surface of a cut MWC. As shown in Fig. 6 (a), the inner surface is smooth and shining, which can reflect visible light with high reflectivity. As shown in Fig. 6(b), the smooth surface is rippled with small terraces and concaves/convexes, due to the deformability and crystalline nature of metal. In view of small area (<5 μm×5 μm), the roughness of most surface is less than 1.2 nm (Fig. 6(c)).

As shown in Fig. 7(a), the optical-path L_OP_ in capillary is decided by incident-angle θ (L_OP_= L_C_/sinθ, where L_C_ is the physical length of capillary). As for Teflon AF capillary filled with DI H_2_O, the incident-angle must be larger than the critical angle of 77.8°, so the L_OP_ is less than 1.02×L_C_ without further enhancement^3^,^6^. While for MWC, confining light inside the capillary does not depend on the refractive-index or incident-angle, so optical-path can be much longer than the length of capillary (L_OP_ » L_C_) by decreasing the incident-angle. As shown in Fig. 7(b), the rippled metal surface could induce light scattering, which can greatly enhance the optical-path.

Thus, for MWC, there are two kinds of optical-path, i.e., straight-light with no reflection (L_OP_ = L_C_), and zigzag-light with multi-reflection (L_OP_ » L_C_) between the sidewalls. According to Beer’s law, the intensity of the transmitted straight- and zigzag-light can be expressed as P_S_×exp(-α×L_C_) and P_Z_×exp(-α×L_OP_), respectively, where the constant α is absorption-coefficient, which is decided solely by ink concentration.

For high concentration ink (e.g., related concentration >1.28 × 10^-5^), the zigzag-light is highly attenuated and its intensity is much lower than that of straight-light, due to the large absorption-coefficient and its much longer optical-path. Thus, the straight-light plays a dominant role in absorbance detection (L_OP_=L_C_), and the AEF keeps a constant value of ~7.0. In contrast, when the absorption-coefficient is decreased with decreasing ink concentration (e.g., related concentration <1.28 × 10^-5^), the intensity of zigzag-light increases more rapidly than that of straight-light, and then zigzag-light begins to play a more important role. Accordingly, AEF can be increased to much larger than 7.0, due to the zigzag optical-path (L_OP_ » L_C_). Accurate light transmitting characteristics of the MWC can be obtained by using the mode theory of waveguide^17^.

Besides the enhancement of optical-path, fast sample switching also contributes to the ultra-low detection limit. Owing to the small volume of MWC (0.16 ml) , the time needed for switching and replacing solutions in the MWC can be less than 20s. As shown in Fig. 5, the minimum detectable value of *A*_*MWC*_ (2.5 × 10^-4^) is 4 times lower than that of *A*_*cuvette*_ (1.0 × 10^-3^). In comparison with the stagnant solution in cuvette, fast switching of flowing solution in capillary could reduce the effect of system noise (such as drifting) on detection precision of absorbance difference. For example, as shown in Fig. 3(b)–(d), the *ΔV* can be easily discriminated from the drifting signals, owing to the fast switching of samples in small volume capillary.

### Application to glucose detection

As shown in Table 2, a series of glucose solutions with various concentrations were prepared with DI H_2_O as solvent. The *colored-* or *blank-samples* were prepared by mixing the glucose solution or DI H_2_O with the chromogenic solution of Glucose Oxidase (GOD) and Peroxidase (POD)^37^, respectively, at a fixed volume ratio of 3:1. Figure 8 shows the optical photograph of the nine *colored-samples* (S2-S10) with glucose concentration ranging from 2.0 mM (on left) to 5.12 nM (on right). The red color decreases with deceasing glucose concentration.

The measurement results of sample 4, 9 and 10 by using the MWC-based photometer are shown in Fig. 9(a)–(c), respectively. As shown in Fig. 9 (c), the measured *ΔV* becomes less stable and its value increases slowly during measurement, because the color of GOD-POD reagent itself (even without adding glucose) can change slowly under illumination. Thus, for the samples with glucose concentration less than 5.12 nM (sample 10), consistent *ΔV* can not be reproducibly measured, because the instability of GOD-POD reagent can no longer be neglected when *ΔV* is small enough. Thus, the detection limit of glucose solution is 5.12 nM, although the corresponding *ΔV* (0.52 μV) is much larger than the noise value (0.03 μV), which indicates that smaller *ΔV* is still detectable. This detection limit can be further improved if employing more stable chromogenic reagent.

The absorbance *A*_*MWC*_ can be calculated with measured *V*_*color*_, *V*_*blank*_ and *V*_*dark*_. The *V*_*dark*_ is −0.068 μV for the photodetector with an amplification-factor of 10^5^. Measurement results of all samples can be founded in supplemental material. For comparison, the glucose samples were also measured by using the spectrophotometer, and the detection limit of measured absorbance *A*_*cuvette*_ reaches 0.64 μM (sample 7) as shown in Fig. 10.

Relationship between the absorbance and concentration was plotted in Fig. 11. In comparison with the cuvette-based spectrophotometer, a 125-fold improvement on detection limit is achieved by using the MWC-based photometer. This improvement is lower than that obtained in red-ink detection, due to the poor stability of GOD-POD reagent. The nonlinear enhancement of absorbance at low concentrations was also observed.

## Conclusion

A MWC-based photometer was developed for ultra-sensitive detection of liquid sample. The optical-path can be greatly enhanced and much longer than the physical length of MWC, because the light scattered by the rippled and smooth metal sidewall can be confined inside the capillary regardless of the incident-angle. For the photometer with a 7 cm long MWC, the detection limit is improved ~3000 fold compared with that of commercial spectrophotometer with 1 cm-cuvette, owing to the novel nonlinear optical-path enhancement as well as fast sample switching, and detecting glucose of a concentration as low as 5.12 nM was realized with conventional GOD-POD reagent. This compact and low-cost photometer would have wide applications in life science and environmental monitor for trace analysis.

## Methods

### Apparatus

As shown in Fig. 1, the MWC-based photometer consists of a 7 cm long MWC (1.7 mm i.d., 3.18 mm o.d., EP grade electropolishing inner surface, SUS316L stainless steel capillary), a 505 nm LED (Thorlabs M505F1) with a lens (the beam spread angle is ~6.6 degree), a gain tunable photodetector (Thorlabs PDB450C), and two T-connectors used for optical coupling and fluid inlet/outlet. The T-connector was fabricated by gluing a transparent quartz plate with a PMMA tube, into which the MWC and a Peek pipe (0.72 mm i.d., 1.6 mm o.d., Vici Valco corp.) were tightly inserted and glued. A three-way valve connected to the inlet Peek pipe is used to switch the inflow samples. The photodetector can convert the received light-power *P* into an amplified voltage signal *N*×*V* (where *V/P* = 1.0 V/W at 1550 nm, and the amplification-factor *N* can be manually tuned in the range of 10^3^-10^7^). *V* is adopted as the output signal rather than *N*×*V* for conciseness.

For comparison, a commercial spectrophotometer (Agilent Technologies Cary 300 Series, equipped with high performance R928 photomultiplier tube) with 1.0 cm cuvette cell was also employed to measure the absorbance of liquid samples.

The inner surface of a cut MWC was investigated by using an optical surface profiler (ZYGO New View 5022) with vertical- and lateral-resolution of 0.1 nm and 0.11 μm, respectively.

A pipette (Finnpipette 1-10 ml, Thermo Fisher Scientific Inc.) was used for pipetting solutions.

### Chemicals and Reagents

All chemicals (analytical grade without further purification) were purchased from Sichuan Maker Biotechnology Co. Ltd. The Glucose Assay Kit includes Glucose Oxidase (GOD), Peroxidase (POD), 4-Aminantipyrine, and phenol, etc. Chromogenic solution was prepared via conventional GOD-POD method^37^.

As shown in Table 2, a series of glucose solutions with various concentrations were prepared with DI H_2_O as solvent by using successive dilution method (details can be found in the supplemental material). The *colored*- or *blank-samples* were prepared by mixing the glucose solution or DI H_2_O with the chromogenic solution, respectively, at a fixed volume ratio of 3:1. All the samples were kept at 37 °C for 10 min in dark before measurement. According to the GOD-POD method, the *colored-sample* would become red with a maximum absorption at wavelength of 505 nm, and the absorbance is nearly proportional to the glucose concentration^37^.

As shown in Table 1, a series of red-ink (Ostrich ink Co., Tianjin, China) solutions were prepared with DI H_2_O as solvent by using successive dilution method.

## Additional Information

**How to cite this article**: Bai, M. *et al.* A compact photometer based on metal-waveguide-capillary: application to detecting glucose of nanomolar concentration. *Sci. Rep.* **5**, 10476; doi: 10.1038/srep10476 (2015).

## Supplementary Material

Supporting Information Supplementary Figures 1-6

## Figures and Tables

**Figure 1:** (**a**) Schematic diagram and (**b**) optical image of the MWC-based photometer.

**Figure 2:** The optical photograph of the red-ink samples.

**Figure 3:** Measurement results of (**a**) sample 6, (**b**) sample 9, (**c**) sample 13 and (**d**) sample14 by using the MWC-based photometer.

**Figure 4:** Measurement results of the red-ink samples by using the spectrophotometer.

**Figure 5:** The relationship between the absorbance and concentration of the red-ink samples.

**Figure 6:** (**a**) The optical image, (**b**) microscopy image and (**c**) optical surface profiler image of inner surface of a cut MWC.

**Figure 7:** Schematic optical reflection in (**a**) Teflon AF capillary filled with DI H_2_O, and (**b**) MWC.

**Figure 8:** The optical photograph of the glucose samples.

**Figure 9:** Measurement results of (**a**) sample 4, (**b**) sample 9 and (**c**) sample 10 by using the MWC-based photometer.

**Figure 10:** Measurement results of glucose samples by using the spectrophotometer.

**Figure 11:** The relationship between the absorbance and concentration of the glucose samples.

**Table 1:** Measurement results of red-ink samples with different concentrations.

**Samples**	**S 4**	**S 5**	**S 6**	**S7**	**S8**	**S9**	**S10**	**S11**	**S12**	**S13**	**S14**
Relative concentration	(1/5)^3^	(1/5)^4^	(1/5)^5^	(1/5)^6^	(1/5)^7^	(1/5)^8^	(1/5)^9^	(1/5)^10^	(1/5)^11^	(1/5)^12^	(1/5)^13^
*V*_*color*_ (μV)	−0.678	−0.678	0.52	5.25	8.65	8.89	9.328	9.218	9.904	9.420	7.960
*V*_*blank*_ (μV)	9.97	9.95	9.80	8.78	9.57	9.12	9.395	9.246	9.917	9.428	7.965
*A*_*MWC*_	3.73	3.72	0.94	0.20	0.041	0.01	0.0029	0.0012	0.00053	0.00034	0.00025
*A*_*cuvette*_	3.40	0.68	0.13	0.027	0.005	0.001	/	/	/	*/*	/

**Table 2:** Measurement results of glucose samples with different concentrations.

**Samples**	**S3**	**S4**	**S5**	**S6**	**S7**	**S8**	**S 9**	**S10**
Concentration	0.4 mM	80 μM	16 μM	3.2 μM	0.64 μM	128 nM	25.6 nM	5.12 nM
*V*_*color*_ (μV)	−0.063	−0.02	3.13	6.5	9.1	10.0	7.74	12.08
*V*_*blank*_ (μV)	10.0	10.6	11.0	9.23	10.4	11.07	8.45	12.6
*A*_*MWC*_	3.255	2.341	0.539	0.15	0.058	0.044	0.038	0.018
*A*_*cuvette*_	1.476	0.385	0.0766	0.019	0.0084	/	/	/
